# Recombinant human PDCD5 (rhPDCD5) protein is protective in a mouse model of multiple sclerosis

**DOI:** 10.1186/s12974-015-0338-0

**Published:** 2015-06-12

**Authors:** Juan Xiao, Wenwei Liu, Yingyu Chen, Wenbin Deng

**Affiliations:** Medical College, Hubei University of Arts and Science, Xiangyang, 441053 China; Department of Immunology, Peking University School of Basic Medical Sciences, Peking University Center for Human Disease Genomics, 38 Xueyuan Road, Beijing, 100191 China; Department of Biochemistry and Molecular Medicine, School of Medicine, University of California-Davis, 2425 Stockton Boulevard, Sacramento, CA 95817 USA

**Keywords:** rhPDCD5, Th1/T17, Multiple sclerosis

## Abstract

**Background:**

In multiple sclerosis (MS) and its widely used animal model, experimental autoimmune encephalomyelitis (EAE), autoreactive T cells contribute importantly to central nervous system (CNS) tissue damage and disease progression. Promoting apoptosis of autoreactive T cells may help eliminate cells responsible for inflammation and may delay disease progression and decrease the frequency and severity of relapse. Programmed cell death 5 (PDCD5) is a protein known to accelerate apoptosis in response to various stimuli. However, the effects of recombinant human PDCD5 (rhPDCD5) on encephalitogenic T cell-mediated inflammation remain unknown.

**Methods:**

We examined the effects of intraperitoneal injection of rhPDCD5 (10 mg/kg) on EAE both prophylactically (started on day 0 post-EAE induction) and therapeutically (started on the onset of EAE disease at day 8), with both of the treatment paradigms being given every other day until day 25. Repeated measures two-way analysis of variance was used for statistical analysis.

**Results:**

We showed that the anti-inflammatory effects of rhPDCD5 were due to a decrease in Th1/Th17 cell frequency, accompanied by a reduction of proinflammatory cytokines, including IFN-γ and IL-17A, and were observed in both prophylactic and therapeutic regimens of rhPDCD5 treatment in EAE mice. Moreover, rhPDCD5-induced apoptosis of myelin-reactive CD4^+^ T cells, along with the upregulation of Bax and downregulation of Bcl-2, and with activated caspase 3.

**Conclusions:**

Our data demonstrate that rhPDCD5 ameliorates the autoimmune CNS disease by inhibiting Th1/Th17 differentiation and inducing apoptosis of predominantly pathogenic T cells. This study provides a novel mechanism to explain the effects of rhPDCD5 on neural inflammation. The work represents a translational demonstration that rhPDCD5 has prophylactic and therapeutic properties in a model of multiple sclerosis.

## Introduction

MS is an inflammatory neurodegenerative disease caused by autoimmune attack against myelin [1]. Impaired apoptotic mechanisms contribute to the production and release of autoreactive T cells that lead to inflammatory demyelination lesions in MS and EAE [2–4]. The mechanisms governing T cell apoptosis are altered by disease [5, 6], and the T cells become more resistant to pro-apoptotic stimuli that trigger caspase activation [7, 8]. The reasons for the decreased susceptibility of activated T cells to apoptosis in MS and EAE are not well understood.

EAE is a CD4^+^ T cell-mediated autoimmune disease model of MS [9, 10]. Both Th1 and Th17 lineages of CD4^+^ T cells are major effector cells responsible for the development of EAE [11–15]. In EAE, T cell apoptosis is thought to be critical for disease recovery [16]. RNAi-mediated knockdown of T-bet, a key regulator of the proinflammatory immune response, ameliorates EAE and limits differentiation of both autoreactive Th1 and Th17 cells [17]. Selective elimination of autoreactive T cells in the CNS of EAE animals is associated with decreased inflammation and reduced disease severity [18]. Administration of apoptosis inhibitors results in impaired recovery and earlier relapse in EAE by suppressing apoptotic death of inflammatory cells in the CNS [19]. Moreover, osteopontin exacerbates EAE symptoms by enhancing the survival of activated T cells and by decreasing levels of pro-apoptotic members of the Bcl-2 family [20]. In contrast, factors increasing the apoptotic sensitivity of T cells reduce disease severity of EAE [21, 22]. Taken together, these findings suggest that promoting the elimination of autoreactive T cells by apoptosis is a possible strategy for treating MS.

Programmed cell death 5 (PDCD5) is initially identified as a gene upregulated in cells undergoing apoptosis [23] and promotes apoptosis in response to various stimuli [24, 25]. In cells undergoing apoptosis, PDCD5 is upregulated and rapidly translocates from the cytoplasm to nucleus [26]. PDCD5 interacts with a histone acetyl transferase, TIP60, and functions as a co-activator to promote apoptosis via the TIP60-p53 signaling pathway [27]. PDCD5 also interacts with p53 and is a positive regulator of p53 gene expression during cell cycle [28]. The recombinant human PDCD5 (rhPDCD5) protein enters cells through clathrin-independent endocytosis and then promotes apoptotic activity [29]. It has been shown that rhPDCD5 sensitizes chondrosarcomas to cisplatin chemotherapy [30], myelogenous leukemia cells to idarubicin (IDR) and aracytidine (Ara-C) chemotherapy [31], and breast cancer cells to paclitaxel chemotherapy [32] by inducing tumor cell apoptosis.

We have shown that PDCD5 transgenic mice develop less severe EAE, accompanied by decreased Th1 and Th17 cells following myelin oligodendrocyte glycoprotein peptide (MOG_35–55_) immunization [33]. In the present study, we examine whether exogenous rhPDCD5 induces apoptosis of myelin-reactive T cells and exerts anti-inflammatory effects against EAE. We show anti-inflammatory activities of prophylactic and therapeutic administrations of rhPDCD5 in EAE mice. Our results demonstrate that both rhPDCD5 regimens decrease Th1/Th17 cell frequency and induce apoptosis of encephalitogenic T cells, indicating that rhPDCD5 is an effective inhibitor of inflammation in an established model of MS in mice.

## Materials and methods

### Chemicals and reagents

Antibodies for detection of the following targets were purchased as indicated: caspase-3 from Cell Signaling Technology; Bax (ab7977) from Abcam; Bcl-2 from BD Biosciences-Pharmingen; and actin from Sigma. Phorbol 12-myristate 13-acetate (PMA), ionomycin, and OVA were purchased from Sigma. Mouse Th1/Th17 phenotyping kit and Perm/Fix solution were purchased from BD Biosciences (USA). IFN-γ and IL-17A ELISA kits were obtained from eBioscience (USA). FITC-anti-CD4 was obtained from Sungene Biotech (Tianjin, china). The MOG35-55 peptide (MEVGWYRSPFSRVVHLYRNGK) was synthesized by Chinese Peptide Company (Hangzhou, China). DyLight 800/DyLight 680-conjugated secondary antibodies against mouse or rabbit IgG were purchased from Rockland Immunochemicals (USA). Recombinant human PDCD5 protein was supplied by Beijing Biosea Biotechnology Co. The endotoxin activity of the rhPDCD5 protein received was <10 EU/mg as detected using the limulus amebocyte lysate assay, and the purity of the rhPDCD5 protein was >95 %.

### Induction, clinical evaluation, and treatment protocols of EAE

C57BL/6 mice were bred at the Experimental Animal Center, Peking University Health Sciences Center (Beijing, China). All experimental procedures and protocols were approved by the Peking University Animal Ethics Committee and were performed in accordance with the institutional guidelines and regulations.

EAE was induced by MOG_35–55_ in female mice used between 8 and 10 weeks of age. Briefly, each mouse was immunized subcutaneously with 300 μg of MOG_35–55_ emulsified with an equal volume of complete Freund’s adjuvant (CFA, total 300 mg of *Mycobacterium tuberculosis*, strain H37RA, Difco, USA) and then injected to the caudal vein with 200 ng of pertussis toxin (dissolved in 200-μl PBS, List Biological Laboratories, USA) at the time of immunization and 2 days later. Mice were examined for clinical scoring daily by the same, blind investigator for 25 days after immunization. Neurological assessments were reported using a 5-point standardized rating scale to evaluate motor deficit as follows: 0, no deficit; 1, tail paralysis; 2, incomplete hind limb paralysis; 3, complete hind limb paralysis; 4, complete hind limb paralysis and partial forelimb paralysis; 5, moribund state or death. Scoring was performed in a blinded fashion.

OVA or rhPDCD5 was dissolved in PBS made up to 2 mg/ml. Prophylactic treatment with rhPDCD5 (10 mg/kg, injected intraperitoneally, i.p.) or OVA (10 mg/kg, i.p.) started on day 0 post-EAE induction and continued every other day until day 25. Therapeutic treatment with rhPDCD5 (10 mg/kg, i.p.) or OVA (10 mg/kg, i.p.) started at the onset of EAE disease (day 8 was the average day of onset of disease) and was given every other day until day 25.

For adoptive transfer of EAE, donor mice were primed by immunization with MOG_35–55_ emulsified with CFA. After 12 days post-immunization, draining lymph node (DLN) lymphocytes and splenocytes were harvested and cultured at 5 × 10^6^/ml in RPMI 1640 for 48 h with 20 μg/ml MOG_35–55_ together with rhPDCD5 (20 μg/ml), and then CD4^+^ T cells were isolated. Recipient mice were sublethally irradiated, then 3 × 10^6^/ml CD4^+^ T cells were transferred intravenously to recipient mice, and pertussis toxin (200 ng) was injected at days 0 and 2 post-CD4^+^ T cell transfer.

### Histological examination

Histological analysis was performed on spinal cords obtained from EAE treated with rhPDCD5 and OVA at day 25 after immunization. Following anesthesia with intraperitoneal administration of pentobarbital, each mouse was perfused with 4 % paraformaldehyde in 0.1 M phosphate buffer. Each spinal cord was carefully removed and immersed in the same fixative. The cervical, thoracic, and lumbar segments of each spinal cord were embedded in paraffin. Five-mm-thick sections were prepared and stained with hematoxylin-eosin (H&E). Semiquantitative histological evaluation for inflammation was scored in a blinded fashion as follows: 0, no inflammation; 1, immune cellular infiltration only in the perivascular area and meninges; 2, mild cellular infiltration in parenchyma; 3, moderate cellular infiltration in parenchyma; 4, severe cellular infiltration in parenchyma.

### Flow cytometry analysis

The DLNs from EAE mice treated with rhPDCD5 and OVA were harvested, and a single cell suspension was prepared. To quantify the number of Th1/Th17 cells, cells were stimulated with PMA and ionomycin in the presence of brefeldin A for 5 h. Subsequently, cells were surface-stained with anti CD4-FITC, permeabilized with Perm/Fix solution and stained with anti-IFN-γ-PE and anti-IL-17A-PE. Isotype-matched IgG was used as a negative control. The stained cells were analyzed by FACSCalibur using CellQuest software (BD Biosciences, USA). For detection of apoptosis, lymphocytes from DLNs of EAE mice were harvested and stimulated with or without of 20 μg/ml of MOG_35–55_ peptide. After 48 h, cells were collected and stained with anti-CD4-PE/AnnexinV-FITC, and percentages of CD4^+^ Annexin V^+^ cells were analyzed by flow cytometry. For detecting the promoting apoptosis effect of rhPDCD5 in vitro, lymphocytes from DLNs of EAE mice were stimulated with MOG_35–55_ and increasing concentration of rhPDCD5. After 48 h, cells were stained with anti-CD4-PE/AnnexinV-FITC, and percentages of Annexin V^+^ cells gated on CD4^+^ T cells were analyzed by flow cytometry.

### Lymphocyte proliferation assay and detection of cytokines in the supernatant and serum

To investigate differences in lymphocyte responses to MOG_35–55_ between OVA and rhPDCD5-treated EAE mice, lymphocytes from DLNs at day 25 were seeded at 5 × 10^5^ cells/well in 96-well plates with RPMI 1640 containing 10 % fetal calf serum (FCS) and stimulated with or without 20 μg/ml of MOG_35–55_ peptide. After 48 h, cells were pulsed with 1 μCi/well [^3^H]-thymidine (MP Biomedicals, USA) and incubated for an additional 8 h. The results are expressed as mean [^3^H] thymidine incorporation (cpm) ± SEM. For detecting cytokines in culture supernatants, lymphocytes were treated as described above. Concentrations of cytokines in the cell supernatant were measured using ELISA kit according to the manufacturer’s instruction. The cytokine concentration in individual mouse serum samples was also detected with the same method.

### Western blot analysis

For experiments of Western blot analysis, lymphocytes from DLNs at day 25 were collected and lysed in lysis buffer (300 mM NaCl, 50 mM Tris pH 8.0, 0.4 % NP-40, 10 mM MgCl_2_, and 2.5 mM CaCl_2_) supplemented with protease inhibitors (Complete mini EDTA-free; Roche Diagnostics, Mannheim, Germany). After centrifugation, the supernatant was measured using the BCA protein assay reagent (Pierce, Rockford, IL, USA). Then, 1 μg of total cell extract protein was loaded onto 12.5 % SDS-PAGE, transferred to nitrocellulose membrane (Amersham Pharmacia Biotech, Little Chalfont, UK), blocked by incubation with 5 % non-fat milk in TBS-T buffer (10 mM Tris–HCl, pH 7.4, 150 mM NaCl, and 0.1 % Tween-20) for 1 h, and blotted against the different proteins using specific antibodies: anti-caspase-3, anti-Bax, anti-Bcl-2, and anti-actin. After washings with TBS, the protein bands were visualized using DyLight 800/DyLight 680-conjugated secondary antibodies, and the infrared fluorescence image was obtained using an Odyssey infrared imaging system (LI-COR Biosciences, USA).

### Quantitative RT-PCR analysis of PDCD5 expression

Total RNA was extracted from DLNs using Trizol according to the manufacturer’s instructions, and 10 μg RNA was reverse-transcribed to cDNA using the cDNA synthesis kit. PCR was performed using *PDCD5* specific primers (5′-CCGAAGCGATTCCAACCGA-3′ and 5′-CTGTCCTAGACACTGCTCCG-3′) to generate a 517 bp product over 35 cycles and *GAPDH* specific primers (5′-CAAGGTCATCCATGACAACTTTG-3′ and 5′-GTCCACCACCCTGTTGCTGTAG-3′) to generate a 496 bp product over 25 cycles of 95 °C for 3 min, 95 °C for 30 s, 58 °C for 30 s, 72 °C for 30 s and 72 °C for 5 min.

### Statistical analysis

For comparisons of the clinical scores of EAE between the OVA- and rhPDCD5-treated animals, repeated measures two-way analysis of variance (ANOVA) followed by Bonferroni post hoc tests were performed to compare replicate by time. Differences in cell frequency and cytokine production between OVA and rhPDCD5-treated mice were evaluated with Student *t*-test. A value of *p* < 0.05 was considered significant.

## Results

### rhPDCD5 treatment attenuates EAE development and protects against spinal cord destruction

C57BL/6 mice were immunized as described in Materials and methods. Ovalbumin (OVA, serving as a negative control) or rhPDCD5 was injected intraperitoneally (i.p.) to each mouse every other day. Mice treated with rhPDCD5 every other day starting at day 0 on the onset of disease induction showed a delayed disease onset and developed less severe EAE than control mice treated by OVA (Fig. 1a). rhPDCD5 injected therapeutically every other day, starting at the onset of EAE disease symptoms (day 8), developed a similar degree of EAE from day 8 to 14 but a faster recovery compared with that seen in OVA-treated EAE mice (Fig. 1b). Histological examinations of the spinal cord tissue collected at day 25 after immunization revealed that minimal lymphocyte infiltration was found in the CNS of mice treated with rhPDCD5 both prophylactically (Fig. 1c) and therapeutically (Fig. 1d), as compared to OVA-treated mice, and the effects of the prophylactic rhPDCD5 regimen were better than the therapeutic regimen.

**Fig. 1:** rhPDCD5 treatment attenuates EAE development and protects spinal cord destruction. EAE mice treated with OVA or rhPDCD5 (10 mg/kg i.p.) **a** prophylactically every other day starting on day 0 following EAE induction and **b** therapeutically every other day from onset of EAE disease (day 8) were monitored daily for mean clinical score. Three independent experiments were performed. Data are means ± SEM from mice treated with OVA (*n* = 10) or rhPDCD5 (*n* = 10). Statistical analysis was performed using repeated measures two-way ANOVA followed by Bonferroni post hoc tests to compare replicate by time. *P < 0.05. **c**, **d** Representative microscopic photographs of spinal cord and semiquantitative histological evaluation for inflammation in EAE mice treated with OVA or rhPDCD5 (10 mg/kg, i.p.) prophylactically and therapeutically stained with H&E are shown. *P < 0.05, **P < 0.005

### rhPDCD5 treatment inhibits IFN-γ and IL-17A production in EAE mice

To investigate the immunological mechanisms associated with the reduced severity of EAE in the rhPDCD5-treated mice, serum samples and DLNs were collected at 25 days after immunization. Cytokine levels in the serum samples were measured by ELISA. Both prophylactic and therapeutic rhPDCD5 treatment of EAE mice produced significantly reduced amounts of serum IFN-γ and IL-17A compared with OVA-treated EAE mice (Fig. 2a, b). We then examined the cytokine production by the DLN cells ex vivo. Single cell suspensions were cultured in the presence or absence of MOG_35–55_ for 48 h, and the supernatants were harvested and analyzed by ELISA for IFN-γ and IL-17A. Cells from EAE mice treated with rhPDCD5 prophylactically and therapeutically produced significantly less IFN-γ and IL-17A in response to MOG_35–55_ compared with cells from OVA-treated mice (Fig. 2c, d). These results therefore indicate that rhPDCD5 promotes downregulation of the inflammatory Th1/Th17 response.

**Fig. 2:** Levels of IFN-γ and IL-17A are downregulated in EAE mice treated with rhPDCD5. **a**, **b** Serum samples were collected from mice treated with OVA or rhPDCD5 prophylactically and therapeutically on day 25 after immunization, and cytokine concentrations were determined by ELISA. Data are means ± SEM (*n* = 10). **c**, **d** Draining lymph node cells were obtained from indicated mice and cultured with or without MOG_35–55_ (20 μg/ml) for 48 h, and the cytokine levels in the culture supernatants were determined by ELISA. Data are means ± SEM (*n* = 10). *P < 0.05, **P < 0.005

### rhPDCD5 treatment reduces Th1/Th17 response in vivo

Inflammatory T cells such as Th1/Th17 cells are thought to play a critical role in the development of EAE. Next, we examined the cellular phenotypes of EAE mice treated with rhPDCD5. Single cell suspensions were prepared from the DLNs of EAE mice 25 day after immunization as described above and stained for cell surface and intracellular markers by FACS. Consistent with the cytokine profile observed above, there was a significant reduction in the frequency of IFN-γ^+^ and IL-17A^+^ cells in the DLNs from EAE mice treated with rhPDCD5 prophylactically (Fig. 3a, b) and therapeutically (Fig. 3c, d) compared with mice treated by OVA. PDCD5 transgenic mice have increased numbers of Foxp3^+^ CD4^+^ regulatory T cells, which protect the mice from EAE [33]. We thus examined whether the recombinant protein rhPDCD5 protects via regulatory T cells, and our results showed that there was no apparent increase in the number and proportion of regulatory T cells during the EAE course, indicating that it is unlikely that the reduced clinical scores of EAE mice treated with rhPDCD5 protein were due to the enhanced regulatory T cells response. Taken together, our data suggest that in vivo rhPDCD5 ameliorates EAE through downregulating the population of inflammatory Th1/Th17 cells.

**Fig. 3:** rhPDCD5 treatment reduces Th1/Th17 response in EAE mice in vivo. **a**, **c** DLN cells were collected from EAE mice treated with OVA or rhPDCD5 (10 mg/kg i.p.) prophylactically and therapeutically at day 25 after immunization and stimulated with PMA plus ionomycin in the presence of brefeldin A for 4 h. CD4^+^IFN-γ^+^ T cells and CD4^+^IL-17A^+^ cells were measured by flow cytometry. **b**, **d** Percentages of CD4^+^IFN-γ^+^ T cells and CD4^+^IL-17A^+^ T cells are shown as means ± SEM (n = 10). *P < 0.05, **P < 0.005

### rhPDCD5 inhibits proliferation of lymphocytes and induces apoptosis of MOG_35–55_ specific CD4^+^ T cells in vivo

Lymphocyte responses to MOG_35–55_ in DLNs from mice treated with OVA and rhPDCD5 prophylactically and therapeutically are shown in Fig. 4a, b. We observed that [^3^H]-thymidine uptake was significantly lower in cells from mice treated with rhPDCD5 prophylactically and therapeutically in vivo, and there was no significant difference in the medium controls between them. This experiment indicates that pretreatment with rhPDCD5 in vivo inhibits the lymphocyte proliferation activated by MOG_35–55_.

**Fig. 4:** rhPDCD5 inhibits lymphocyte proliferation to MOG. Lymphocytes were obtained from DLNs in EAE mice treated with OVA or rhPDCD5 prophylactically (**a**) and therapeutically (**b**) at day 25 after immunization, cultured with or without MOG_35–55_ (20 μg/ml) for 48 h. Cell proliferation was determined by the uptake of [^3^H] incorporation. Data are means ± SEM (*n* = 8). ***P < 0.0005

Given the pro-apoptotic function of PDCD5, we next monitored CD4^+^ T cell apoptosis using FITC-Annexin V staining and flow cytometry analysis. Single cell suspensions were prepared from the DLNs of EAE mice at day 25 after immunization and stained for CD4 and AV by FACS. There was a significant increase in the frequency of CD4^+^AV^+^ cells in the DLNs from EAE mice treated with rhPDCD5 prophylactically (Fig. 5a, b) and therapeutically (Fig. 5c, d) compared with mice treated by OVA. Without MOG_35–55_ stimulation, the percentage of CD4^+^ T cell apoptosis was not different between EAE mice treated with OVA or rhPDCD5. In normal mice without EAE, rhPDCD5 did not induce apoptosis and did not alter the number of lymphocytes. RhPDCD5 treatment only induced apoptosis of MOG-activated T cells but not normal T cells. It is likely that rhPDCD5-induced cell death may explain the lower level of inflammation and downregulation of Th1/Th17 cells in EAE mice treated with rhPDCD5 prophylactically and therapeutically in vivo.

**Fig. 5:** rhPDCD5 induces apoptosis of MOG-stimulated T cells in vivo. **a**, **c** Lymphocytes were obtained from DLNs in EAE mice treated with OVA or rhPDCD5 prophylactically and therapeutically at day 25 after immunization, cultured with or without MOG_35–55_ (20 μg/ml) for 48 h. Cellular apoptosis was analyzed by FITC-Annexin V plus anti-CD4-PE staining and flow cytometry. **b**, **d** Percentages of CD4^+^AV^+^ T cells are shown as means ± SEM (*n* = 10). **P < 0.005

### rhPDCD5 induces activation of caspase-3, enhances the expression of Bax, and suppresses the expression of Bcl-2

To address the mechanism of rhPDCD5-induced cell death, cells were extracted from DLNs at day 25 post immunization and analyzed by Western blotting the expression of Bcl-2, Bax and activated caspase-3. As shown in Fig 6a, b, lower levels of Bcl-2 but increased levels of Bax and activated caspase-3 were detected in lymphocytes pretreated with rhPDCD5 prophylactically and therapeutically in vivo.

**Fig. 6:** The expression of caspase-3, BAX, and BCL-2 in EAE mice. **a**, **b** Lymphocytes were collected from DLNs in EAE mice treated with OVA or rhPDCD5 (10 mg/kg i.p.) prophylactically and therapeutically at day 25 after immunization. Cell lysate was examined for the expression of procaspase-3 (inactive form), cleaved caspase 3 (active form), BAX, and BCL-2 by Western blot analysis. Actin was used as a housekeeping protein, and the gels have been run under the same experimental conditions. The relative levels of procaspase 3/cleaved caspase 3 were quantified by densitometric analysis and normalized with Actin. Data are means ± SEM (*n* = 4). Statistical differences were evaluated with Student *t*-test. *P < 0.05

### rhPDCD5 induces apoptosis of MOG_35–55_ specific CD4^+^ T cells

Single cell suspensions from DLNs of EAE mice at day 12 after immunization were stimulated with MOG_35–55_ and increasing concentrations of rhPDCD5 for 48 h. Cells were then stained with CD4 and AV by FACS. A dose-dependent effect was seen in rhPDCD5-induced MOG-specific apoptosis of CD4^+^ T cells (Fig. 7a). The same treated lymphocytes were collected and then examined for the expression of PDCD5 by Western blot analysis. As shown in Fig. 7b, the expression of PDCD5 mRNA and protein level increased along with the increase of cell apoptosis, indicating that endogenous PDCD5 is upregulated when lymphocytes undergo apoptosis.

**Fig. 7:** rhPDCD5 induces apoptosis of MOG-specific T cells. **a** Apoptosis of CD4^+^ T cells was determined and quantified by the percentage of AV positive cells showing an increase in a dose-dependent manner, and representative histograms are shown. **b** Lymphocytes treated with rhPDCD5 were examined the expression of PDCD5 mRNA and protein levels by RT-PCR and Western blot analysis. Gels have been run under the same experimental conditions. **c** DLN lymphocytes and splenocytes isolated from donor mice 12 days post-immunization were re-stimulated with MOG and rhPDCD5, and 3 × 10^6^/ml CD4^+^ T cells were transferred into irradiated naïve mice to induce passive EAE. Mice were then monitored daily for mean clinical score. Two independent adoptive transfer experiments were performed. Data are means ± SEM from mice treated with MOG (*n* = 8) or MOG+ rhPDCD5 (*n* = 8). Statistical analysis was performed using repeated measures two-way ANOVA followed by Bonferroni post hoc tests to compare replicate by time. *P < 0.05

To directly demonstrate whether rhPDCD5 could induce apoptosis of MOG-reactive CD4^+^ T, CD4^+^ T cells isolated from MOG-immunized donor mice were re-stimulated with MOG together with rhPDCD5 in vitro and then adoptively transferred to naïve mice to induce passive EAE. Notably, rhPDCD5 (20 μg/ml) pretreated CD4^+^ T cells induced a less severe EAE symptom than CD4^+^ T cells re-stimulated by MOG only (Fig. 7c). These results indicate that rhPDCD5 acts by increasing apoptosis of MOG-reactive CD4^+^ T cells.

## Discussion

Data presented in this study demonstrate that treatment of EAE mice with rhPDCD5 shows benefits at both clinical and pathological levels. The protection against EAE is not only due to downregulation of Th1/Th17 cells but also attributable to higher levels of activation-induced cell death in T cells, with both prophylactic and therapeutic rhPDCD5 treatment regimens in vivo. Furthermore, we show that the expression of Bax and caspase 3 is increased and expression of Bcl-2 is decreased in lymphocytes treated by rhPDCD5 in vivo. In addition, rhPDCD5 induces apoptosis of myelin-specific CD4^+^ T cells in vitro.

EAE is a well-known model of MS, the most common chronic neuroinflammatory, demyelinating disease of the CNS in humans. In the past, EAE was considered to be a Th1-driven disease. However, the discovery of a third major helper T cell subclass, called Th17 cells, has substantially increased our understanding of the cellular basis of EAE pathogenesis [11, 34]. Both Th1 and Th17 cells have been shown to be capable of driving EAE, but neither cell type can exclusively induce pathogenesis of the same extent without a contribution from the other [35–37]. In the context of the present study, it is likely that the reduced clinical symptom and pathology in EAE mice treated with rhPDCD5 prophylactically and therapeutically is due to the decreased Th1/Th17 cell frequency, accompanied by a reduction of pro-inflammatory cytokines in the serum. PDCD5 has been implicated in the downregulation of Th1 and Th17 cells in PDCD5 transgenic mice [33]. This study is the first to show that exogenous recombinant human PDCD5 protein can induce the downregulation of Th1/Th17 cells in vivo. The polarization of naïve T cells into Th1/Th17 cells depends on the cytokine milieu in the tissue. Whether rhPDCD5 affects the cytokine milieu or directly enters the lymphocytes to inhibit the differentiation of Th1/Th17 remains unclear.

During the course of EAE, inflammatory lymphocytes enter the CNS and elicit variable degrees of demyelination and inflammation [38]. The ongoing inflammation is manifested by clinical signs, such as paresis and paralysis of the limbs. In the EAE mouse model, factors leading to increased apoptosis of activated T cells have been shown to decrease disease severity [21, 22], while factors that decrease the apoptosis of activated T cells increase disease severity [18, 19]. At any time during EAE, the magnitude of T cell responses against myelin antigen involves the balance between an increasing number of myelin-specific lymphocytes due to cell division and loss of T cells by activation-induced cell death. During EAE recovery, apoptosis is a leading mechanism for the clearance of CNS infiltrating cells [39]. Our experiments show that rhPDCD5 is involved in the apoptosis of activated CD4^+^ lymphocytes as we observe an increase in the proportion of MOG_35–55_ activated CD4^+^ lymphocytes undergoing apoptosis in rhPDCD5-treated mice compared to OVA-treated mice. Moreover, rhPDCD5 induces apoptosis of myelin-specific T cells in a dose-dependent manner in vitro, accompanied by upregulation of endogenous PDCD5 in lymphocytes, indicating that PDCD5 is upregulated when lymphocytes undergo apoptosis. Whether rhPDCD5 selectively enters lymphocytes during EAE is an intriguing question that warrants further investigation. It has been shown that exogenous rhPDCD5 promotes apoptosis in a number of tumor cells [23, 30–32, 40], but to our knowledge, this study is the first to demonstrate that rhPDCD5 induces apoptosis of antigen-activated mature T lymphocytes.

Apoptosis is a developmentally and physiologically critical process that is tightly regulated by the coordinated action of diverse extracellular cues and intracellular signaling molecules. Specifically, the Bcl-2 family of proteins has been shown to play important roles in several different pathways affected by apoptosis, with the ratio of Bax/Bcl-2 being critical for the induction of apoptosis. Bcl-2 is an anti-apoptotic protein that prevents the initiation of apoptosis by blocking the efflux of cytochrome c from mitochondria [41]. Overexpression of Bcl-2 in lymphocytes suppresses apoptosis and promotes development of T and B cells [42]. Furthermore, it has been shown that overexpression of Bcl-2 delays caspase-3 activation and rescues cerebellar degeneration in prion-deficient mice [43]. Caspase-3 is a crucial mediator that catalyzes the cleavage of several key proteins to trigger apoptosis [44]. Using Western blot analysis of lymphocytes of EAE mice, we showed that expression of Bax and activated caspase-3 was increased but expression of Bcl-2 was decreased in lymphocytes treated with rhPDCD5 in vivo, in agreement with an earlier report [30].

In summary, our study demonstrates that rhPDCD5 has a protective role in EAE, and rhPDCD5 is a potential therapeutic agent for MS. The beneficial effects of rhPDCD5 are associated with downregulation of Th1/Th17 response and activation-induced T cell death. For future studies, it would be interesting to further investigate the exact function of rhPDCD5 in the CNS, the direct effect of rhPDCD5 on demyelination and remyelination, and the precise mechanism by which rhPDCD5 acts in the experimental model of MS.
